The article "Combined Case of Blood-Injury-Injection Phobia and Social Phobia: Behavior Therapy Management and Effectiveness through Tilt Test" was retracted in 2016. Reasons: plagiarism; overlap with other authors' work; concerns about the citations.

# Combined Case of Blood-Injury-Injection Phobia and Social Phobia: Behavior Therapy Management and Effectiveness through Tilt Test

**DOI:** 10.1155/2012/368039

**Published:** 2012-12-13

**Authors:** Fotini Ferenidou, Theodoros Chalimourdas, Velissarios Antonakis, Nikolaos Vaidakis, Georgios Papadimitriou

**Affiliations:** ^1^1st Department of Psychiatry, Eginition Hospital, University of Athens Medical School, Vas. Sofias 72, 11528 Athens, Greece; ^2^1st Cardiology Clinic, Hippokration Hospital, University of Athens Medical School, Vas. Sofias 114, 11527 Athens, Greece

## Abstract

The efficacy of behavior therapy based mainly on real-life exposure situations as well as applied tension was examined for a combined case of blood-injury-injection (BII) phobia and social anxiety disorder. Treatment involved 28 behavior therapy sessions, while applied tension technique was also described and practiced. The specific contribution of social skills techniques, fantasy, and real-life situations exposure was examined in a single case design. The subject was a 39-year-old male with anxiety symptoms when confronting an audience, as well as symptoms of the autonomic nervous system (bradycardia and syncope), which were better explained by BII. All self-report measures regarding fear, social phobia, and anxiety were reduced after behavior therapy and remained maintained at followup, while BII decreased further after applied tension techniques. The contribution of behavior therapy to the overall outcome of the case is considered significant for many reasons that are discussed in the pape.

## 1. Introduction

Blood-injury-injection phobia (BII) is quite a common phobia. Estimates of lifetime prevalence of BII phobia range 3.5% for men and women [1] to as high as 4.9% for women [2], and unlike individuals with other specific phobias, 75% of those with BII phobia report a history of fainting in response to phobic stimuli. 

 The most outstanding characteristic of blood phobics is their unique physiological pattern when confronted with the phobic stimuli. The fainting response is characterized as a vasovagal syncope and has been described in the literature as a two-phase, or biphasic (also called diphasic) response to BII stimuli [3, 4]. The initial phase involves an increase in heart rate and blood pressure as is typical of the fight-flight component of an anxiety response [5], whereas the second phase is characterized by bradycardia and hypotension leading to reduced cerebral blood flow and ultimately fainting [4], although this pattern is not always observed [6].

 Fainting in response to BII stimuli is a significant source of concern for many patients suffering from blood phobia and can aggravate avoidance. According to the DSM-IV-TR [7], the fear that is cued by the presence or anticipation of the feared stimulus (e.g., receiving an injection or seeing blood) is deemed unreasonable and excessive. If the situation is not avoided altogether, the afflicted person endures the phobic object (e.g., blood) or situation (e.g., going to the doctor) with intense anxiety or distress. Consequently, significant interference with the person's normal routine, including occupational and social functioning, is observed and is a necessary diagnostic criterion [8]. The treatment technique generally recognized as efficacious for BII phobia is Applied Tension (AT), which combines a muscle tension technique with in vivo exposure [6, 9, 10]. The tension technique utilizes repeated tense and release sequences of the skeletal muscles to counteract cardiovascular and autonomic changes implicated in BII-related syncope. Versions of this technique have been used for some time for combating orthostatic hypotension in patients as well as fainting in various settings such as blood donation [11–14]. 

 Kozak and Montgomery [15] are generally regarded as the first to have devised AT as a behavioral treatment strategy for BII phobia. Their aim was to target the syncopal episode rather than the initial anxious arousal, which is typically observed as the first stage of the biphasic response. The tensing of skeletal muscles involved in this technique led to increases in blood pressure and heart rate, and was thereby thought to counteract the two major autonomic phenomena involved in the vasovagal syncope: hypotension through peripheral vasodilation and bradycardia by massive vagal excitation. In addition, skeletal muscle tension (particularly in the extremities) promoted increased blood flow to the heart and brain, thereby preventing the fainting response [16].

 Social Anxiety Disorder (SAD) or Social Phobia, as defined in DSM-IV-TR [7], is a marked and persistent fear of one or more social or performance situations in which the person is exposed to unfamiliar people or to possible scrutiny by others. The individual fears that he or she will act in a way (or show anxiety symptoms) that will be humiliating or embarrassing. Activities such as meetings or interactions with strangers, attending social gatherings, formal presentations, and those requiring assertive behavior are commonly feared by individuals with social phobia [17]. The recent National Comorbidity Survey [18] reported a lifetime prevalence of 13.3% for social phobia and its prevalence appears to be increasing [19]. Social phobia is highly comorbid with other anxiety disorders, depression, and substance abuse, and it significantly increases the risk for these disorders [20]. It runs a chronic course and is associated with significant impairments in functioning and overall quality of life, as well as an increased risk of suicidal ideation and attempts [21–24].

 Research on SAD has demonstrated that cognitive, behavioral, and physiological components are all present and interact in the presentation of this disorder [25]. For instance, individuals with SAD tend to engage in more self-monitoring of their own behavior, focus on potential threats, believe that individuals will notice their anxiety symptoms and interpret them negatively, and are more likely to perceive their behaviors negatively than individuals without social anxiety [17, 26–28]. Due to the cognitive, behavioral and physiological components of SAD, numerous studies have investigated the efficacy of cognitive-behavioral therapy (CBT) on SAD. In fact, CBT is the most widely used and researched treatment for SAD [29]. Research has consistently shown CBT to be an efficacious treatment for SAD when administered either individually or in a group format [30–32]. 

 In order to make a good match between the phobic patient and treatment method one can scrutinize the available techniques and decide which of the three anxiety components each method is focused on. So, for example, social skills training, reinforced practice, flooding, modeling, and contact-desensitization can be viewed as focusing on the behavioral component. Techniques such as stress-inoculation training and systematic rational restructuring concentrate on the cognitive component, while the physiological component is the primary target for relaxation methods (e.g., applied relaxation), anxiety management training, systematic desensitization and biofeedback. Naturally, some of the techniques contain aspects of more than one component but the above categorization is based on each technique's primary characteristic [33].

The article "Combined Case of Blood-Injury-Injection Phobia and Social Phobia: Behavior Therapy Management and Effectiveness through Tilt Test" was retracted in 2016. Reasons: plagiarism; overlap with other authors' work; concerns about the citations.

## 2. Case Presentation

### 2.1. Subject

The subject was—at the beginning of treatment—a 39-year-old male, married with one child. He was working as a Lecturer at the University and was the third child of a 5-member family. His parents were divorced since 1985, when the patient was 13 years old. He reported a prior history of anxiety symptoms during his lectures in front of an audience, which were often accompanied by syncope and serious injuries. Since syncope cannot be explained by social phobia, it was considered necessary to perform an autonomous nervous system exam. Tilt test was performed and found abnormal results (quite important reduce in heart rate). Additionally, several medical history facts (drop in blood pressure when being present in procedures that included blood) substantiated BII phobia. No prior psychiatric or medical history was reported.

 Regarding his family history, his father was hospitalized in a psychiatric institution twice, involuntarily, when the patient was 7 and 15 years old. Furthermore, his uncle—his father's brother—was referred as “the village's crazy guy”, showing quite often “abnormal” behavior. Equivalent mental problems were referred regarding his paternal grandmother (behavioral problems) and his other uncle (from his mother's side-alcoholic and violent). His mother reported BII, which she managed to get over after her first baby delivery. The subject was going under psychoanalytic psychotherapy for the last two years, with mild improvement. He had never received any pharmacological compounds regarding his problem, before or during behavior therapy.

### 2.2. Measures

The State-Trait Anxiety Inventory [34] is comprised of 40 items divided evenly between state anxiety and trait anxiety. The authors reported reliability for trait anxiety was 0.81; as expected, figures were lower for state anxiety (0.40). Internal consistency ranges between 0.83 and 0.92.

 The Fear Questionnaire [35] is a one-page self-rating form described to monitor change in phobic patients. The form yields four scores: main phobia, global phobia, total phobia, and anxiety-depression. The total phobia score is composed of agoraphobia, social, and blood-injury subgroups. The form is short, reliable, and valid. 

 The Liebowitz Social Anxiety Scale (LSAS) is the first clinician-rating scale developed for the assessment of social phobia [36] and was designed to assess the range of social interaction and performance situations that individuals with social phobia may fear and/or avoid [37]. Its 24 items are divided into two subscales that address social interactional (11 items) and performance (13 items) situations. The clinician asks the patient to rate fear and avoidance during the past week on 0–3 Likert-type scales; however, the clinician is given latitude to question the patient's responses and adjust the ratings accordingly. Thus, the LSAS provides six subscale scores: total fear, fear of social interaction, fear of performance, total avoidance, avoidance of social interaction, and avoidance of performance. An overall total score is often calculated by summing the total fear and total avoidance scores, and this index is the one most commonly employed in studies of the pharmacotherapy of social phobia.

 The Beck Anxiety Inventory (BAI), created by Beck and Steer, is a 21-item multiple-choice self-report inventory that measures the severity of anxiety in adults and adolescents. Because the items in the BAI describe the emotional, physiological, and cognitive symptoms of anxiety but not depression, it can discriminate anxiety from depression. Each of the items on the BAI is a simple description of a symptom of anxiety in one of its four expressed aspects: (1) subjective (e.g., “unable to relax”), (2) neurophysiologic (e.g., “numbness or tingling”), (3) autonomic (e.g., “feeling hot”), or (4) panic-related (e.g., “fear of losing control”) [38].

 A tilt table test, occasionally called upright tilt testing, is a medical procedure often used to diagnose dysautonomia or syncope. Patients with symptoms of dizziness or lightheadedness, with or without a loss of consciousness (fainting), suspected to be associated with a drop in blood pressure or positional tachycardia are good candidates for this test. The procedure tests for causes of syncope by attempting to cause syncope by having the patient lie flat on a special table or bed while connected to ECG and blood pressure monitors. The table then creates a change in posture from lying to standing [39].

The article "Combined Case of Blood-Injury-Injection Phobia and Social Phobia: Behavior Therapy Management and Effectiveness through Tilt Test" was retracted in 2016. Reasons: plagiarism; overlap with other authors' work; concerns about the citations.

### 2.3. Procedure

The subject was referred to the second author for treatment of social phobia. He underwent 28 weekly behavioral therapy sessions based on exposure to real-life experiences (the total therapy time frame was 7 weeks). Twenty sessions had to do with social phobia management, 8 had to do with BII management and their duration was approximately 45 minutes each. During visits 1 and 2, history taking took place, while during visits 3, 4, and 5 the therapist went through behavioral analysis, psychoeducation and target specification. Behavioral analysis included the stimulants as well as the physical, cognitive, and behavioral reactions that they trigger. Stimulants were his position as an observational subject in front of an audience (during his lectures or when he expresses his opinion), as well as when he faces colleagues that belong to a higher academic level than his. Additionally, pictures and thoughts that had to do with blood seemed to provoke the same reaction. Physical reactions were sweating, muscle tension, tachypnea, dizziness, scotodinia, syncope, while cognitive reactions were thoughts such as: “I am inadequate, I will not make it, I will faint and be ridiculed.” Finally, behavioral reactions (avoidance and coping strategies) had to do with sitting versus standing, avoiding eye contact, not expressing his opinion, whispering instead of speaking out, or even exiting the room. The above-mentioned reactions had a great impact on his job (professional restrictions, thinking of quitting his job) as well as restrictions in his social life.

 During visits 6–9, role playing, relaxation techniques, and imaginable exposure to anxiety stimulants took place, while visits 10–15 included gradual exposure to real-life stimulants. First, exposure took place at his work place, for example, giving difficult lectures in front of a small audience, in front of Ph.D. students or other university teachers that he well knew and gradually in front of professors of higher academic level. The subject received assertiveness training and sessions 15 to 18 included exposure to other situations. He was asked to be loud while talking on the phone, at the super market, to make frequently questions to people he did not know (e.g., on the street) and to even risk feeling shame and losing acceptance from others. 

 Taking into consideration the fact that social phobia alone cannot explain syncope, as well as information from the patient's history, blood-injury-injection (BII) phobia seemed to be also present obstructing behavior therapy. BII—as mentioned above—is usually followed by a two-phase vasovagal response. First, due to the action of the sympathetic nervous system, heart rate, and blood pressure increase, but after a while the parasympathetic nervous system takes action followed by sudden reduce in heartrate and blood pressure. The degree to which the cardiovascular system responses, differentiates patients from healthy population. Bradycardia—as a response to the fearful stimulant—may lead to syncope, while fear is sustained since possible syncope leads to anxiety. Applied tension seems to be an effective treatment for blood phobia [40]. The rationale for applied tension is very simple, and after describing the diphasic pattern the patient is given the following explanation. As the second phase of the diphasic response consists of a rapid drop in BP the cerebral blood flow is also reduced and the patient feels dizzy, and eventually faints. In order to reverse this development the patient needs to learn a coping skill that can be applied quickly and easily in almost any situation. One coping skill that produces an increase in BP and cerebral blood flow is applied tension. This consists of two parts; first learning to tense the gross body muscles, and second learning to identify the earliest signs of the drop in BP, and using these as a cue to apply the tension technique. By being exposed to different blood-injury stimuli under the therapist's supervision, the patient will gradually grow more and more efficient in identifying these early signs and applying the tension [41]. The tension technique was as follows: the patient was instructed to tense the muscles of the arms, the chest, and the legs, and keep tensing until a feeling of warmth is rising in the face (10–20 sec). Then she/he lets go of the tension and returns to the starting level, but does not relax further. After a pause of 20–30 sec the patient does the tension again, and then releases it. This procedure is repeated 5 times, and as homework assignment the patient is instructed to perform 5 tension-release cycles 5 times a day. The technique is supposed to take place in combination with real-life situations and has as a goal reverse of the two-phase vasovagal response. Therefore, syncope is prevented and patient's confidence is reinforced. Sessions 19 and 20 included the above-mentioned information and education, accompanied by special brochures.

 Finally, sessions 21 to 28 included real-life exposure to blood and blood related procedures. Specifically, the patient—together with his therapist—observed blood collection and blood donation procedures in a hospital and came in touch with syringes and needles. He even had his own blood collected, became a blood donor and watched a surgical procedure with success (without feeling any of the previously mentioned symptoms). 

The article "Combined Case of Blood-Injury-Injection Phobia and Social Phobia: Behavior Therapy Management and Effectiveness through Tilt Test" was retracted in 2016. Reasons: plagiarism; overlap with other authors' work; concerns about the citations.

### 2.4. Outcome

 The subject was administered the battery of questionnaires described above just before the beginning of treatment, after the end of treatment (after session 28), and at 6 and 18 months posttreatment. Total results of the questionnaires are presented in Figure 1. The results of the questionnaires separately can be found in Figures 2, 3, 4, and 5. As can be seen, his self-reported fear, social phobia and anxiety were reduced after behavior therapy and were maintained at followup. BII was quite reduced after exposure techniques and applied tension methods. Additionally, tilt test was performed three times during behavior therapy sessions, but was stopped due to important reduce in heart rate. Specifically, it took place at the beginning of therapy (1st session), in the middle (16th session) and in the end of treatment (28th session). The first tilt test was stopped at the first minute due to bradycardia, low blood pressure and syncope. The second tilt test was also stopped during the first minute due to similar symptoms (although syncope did not occur), and the third tilt test was stopped during the 3rd minute due to symptoms of the autonomic nervous system. During the fourth tilt test (18 months posttreatment), patient remained symptom free and hemodynamically stable throughout the whole procedure (20 minutes duration). Finally, BII was quite reduced after exposure techniques and applied tension methods.

## 3. Discussion

 Behavior therapy was successful in reducing this subject's social phobia as well as BII phobia. Although the sole contribution of behavior therapy to his improvement is not possible to determine given the inclusion of psychoanalytic sessions 2 years before, the contribution of behavior therapy to the overall outcome is considered significant for many reasons. First, his self-reported social phobia, blood injury phobia and social anxiety on all measures as well as general symptoms of anxiety (as measured by the Beck Anxiety Inventory) decreased further following behavior therapy. Second, he was able to take over as a president of a control committee on organic foods, a responsibility he used to avoid before, because of the stress it provoked him. Third, he was a candidate of the workforce committee of his workplace (he had to introduce himself to many people, talk about himself and his achievements), where he was finally elected as president. Fourth, he represented many times abroad the Ministry he was working for with quite success.

 His own comments regarding behavior therapy and exposure in particular were as follows: “The method was liberating, since I realized that I was trapped in a game where I had to get confirmation from everybody;” “After some (therapy technique) repetitions I felt really free and I realized that true freedom comes when someone is free from his fears.” His comments regarding relaxation included: “The first relaxation experience was amazing. I truly relaxed and realized that it was years since I felt calm and self-concentrated;” “It helped me deal with the anxiety of expecting something, for example, before the beginning of a class I try to practice relaxation techniques in order to deal with the permanent anxiety—which wouldn't let me think clearly—and not overestimate things.” Finally his comments regarding training on assertiveness skills were: “ During class I try—and most of the times I succeed—to be myself without trying to imitate my “serious” professors; the way my body moves, my smooth voice, my low profile and my friendly mood towards students, have a relaxing impact on me since I no more try to be someone else rather than myself;” “ I do not hesitate to admit that I do not know something, which is quite soothing for me since I do not need to know everything.”

 According to the social skills deficit model, people with social anxiety lack important skills to interact effectively with others. Consequently, they experience fewer interpersonal rewards and more punishments, leading them to avoid social interactions when possible, thereby further limiting their ability to acquire effective social skills. Accordingly, comprehensive treatment for social anxiety would provide explicit training to help patients acquire and use appropriate social skills and thereby reverse the negative cycle [42]. Research on SAD has demonstrated that cognitive, behavioral, and physiological components are all present and interact in the presentation of this disorder [25]. To summarize the experimental studies on social phobia in psychiatric patients, one could say that the effects of treatment are rather modest. All the studies reviewed found significant changes on different self-report measures. No consistent results pointing to the superiority of any method studied has emerged and results seem to depend on the anxiety component that is prominent in each patient [33].

 Blood-injury-injection (BII) phobia presents with a unique anxiety response that often involves blood pressure drops and pronounced bradycardia, which can culminate in fainting. Although the current recommended treatment for BII phobia is Applied Tension (AT) surprisingly little empirical evidence is available on the additive efficacy of tension beyond exposure alone. Literature search yielded five controlled treatment studies for BII phobia, all from one research group. Beyond AT, these studies also tested Exposure only (E), Tension only, Applied Relaxation (AR), or a combination of AR and AT. Based on self-reported levels of anxiety, in-session avoidance and fainting, AT was superior over other conditions; however, when considering pre- to posttreatment effect sizes on BII-related questionnaires, E outperformed all other treatments. In addition, AT did not yield better results on physiological measures, and individuals with BII fears improved similarly within studies across treatment groups, regardless of fainting status. Heterogeneity in patient populations (e.g., extent of fainting proneness), differential targeting of BII phobia manifestations, and small sample sizes may explain some of the variability in findings [16]. Although the present case study shows significant results for BII therapy with a combination of blood related procedures exposure and applied tension, further research is needed to determine the efficacy of treatment techniques for BII phobia patients with and without fainting history. 

The article "Combined Case of Blood-Injury-Injection Phobia and Social Phobia: Behavior Therapy Management and Effectiveness through Tilt Test" was retracted in 2016. Reasons: plagiarism; overlap with other authors' work; concerns about the citations.

## Figures and Tables

**Figure 1:** Questionnaires' scores pre- and posttreatment and followup.

**Figure 2:** Marks & Mathews fear Questionnaire pre- and posttreatment and follow up.

**Figure 3:** Liebowitz Social Anxiety Scale (LSAS) pre- and posttreatment and followup.

**Figure 4:** Spielberger State-Trait Anxiety Inventory pre- and posttreatment and follow up.

**Figure 5:** Beck Anxiety Inventory pre- and posttreatment and followup.
